# Colon and rectal surgery for cancer without mechanical bowel preparation: One-center randomized prospective trial

This article has been retracted.

**DOI:** 10.1186/1477-7819-8-35

**Published:** 2010-04-30

**Authors:** Stefano Scabini, Edoardo Rimini, Emanuele Romairone, Renato Scordamaglia, Giampiero Damiani, Davide Pertile, Valter Ferrando

**Affiliations:** 1 Unit of Surgical Oncology, Department of Emato-Oncology, San Martino Hospital, Genoa, Italy

## Abstract

**Background:**

Mechanical bowel preparation is routinely done before colon and rectal surgery, aimed at reducing the risk of postoperative infectious complications. The aim of the study was to assess whether elective colon and rectal surgery can be safely performed without preoperative mechanical bowel preparation.

**Methods:**

Patients undergoing elective colon and rectal resections with primary anastomosis were prospectively randomized into two groups. Group A had mechanical bowel preparation with polyethylene glycol before surgery, and group B had their surgery without preoperative mechanical bowel preparation. Patients were followed up for 30 days for wound, anastomotic, and intra-abdominal infectious complications.

**Results:**

Two hundred forty four patients were included in the study, 120 in group A and 124 in group B. Demographic characteristics, type of surgical procedure and type of anastomosis did not significantly differ between the two groups. There was no difference in the rate of surgical infectious complications between the two groups but the overall infectious complications rate was 20.0% in group A and 11.3% in group B (p .05). Wound infection (p = 0.18), anastomotic leak (p = 0.52), and intra-abdominal abscess (p = 0.36) occurred in 9.2%, 5.8%, and 5.0% versus 4.8%, 4.0%, and 2.4%, respectively. No mechanical bowel preparation seems to be safe also in rectal surgery.

**Conclusions:**

These results suggest that elective colon and rectal surgery may be safely performed without mechanical preparation.

## Background

In the first half of the 20th century, mortality from colon and rectal surgery often exceeded 20%, [1] mainly attributed to sepsis. Modern surgical techniques and improved perioperative care have significantly lowered the mortality rate. Infectious complications, however, still are a major cause of morbidity in colorectal surgery, leading to increased cost, prolonged hospital stay, and occasional mortality [2].

Mechanical bowel preparation is aimed at cleaning the large bowel of fecal content, there by reducing the rate of infectious complications following surgery. Traditionally, bowel cleansing was achieved using enemas in combination with oral laxatives [3]. More recently, oral cathartic agents to induce diarrhea and cleanse the bowel from solid feces were developed. These new bowel preparation agents, such as polyethylene glycol and sodium phosphate, provide superior cleansing compared to the more traditional methods [4-6] and are used by most surgeons in preparation for colorectal surgery [7-9]. The practice of bowel cleansing before colorectal surgery has became a surgical dogma, and primary colonic anastomosis is considered unsafe in the face of an unprepared bowel. There is, however, a paucity of data showing that mechanical bowel preparation by itself, separately from other operative and perioperative measures, actually reduces the rate of infectious complications.

In urgent colon surgery for penetrating trauma, many studies have shown that primary colonic anastomosis is safe even though mechanical bowel preparation is not performed before surgery [10,11]. These data therefore may bring into question the utility of mechanical bowel preparation in elective colon and rectal surgery.

Recently two studies [12,13] show no benefit of mechanical bowel preparation in elective colorectal resection and Bretagnol [14] says that avoid bowel preparation may be associated with reduced postoperative morbidity in elective rectal cancer surgery.

Finally a Cochrane review [15] concluded that there is no statistically significant evidence that patients benefit from bowel preparation, but this study requires further research on patients submitted for elective colorectal surgery in whom bowel continuity is restored, with stratification for colonic and rectal surgery.

The aim of this study was to assess whether elective colon and rectal surgery may be safely performed without preoperative mechanical bowel preparation also considering stratification in patients underwent at colon or rectal surgery.

## Methods

Patients undergoing elective colon and rectal surgery with primary anastomosis in our Oncologic Unit Surgery between july 2005 and september 2009 were prospectively randomized by individual computer-generated randomization into two groups. Patients in Group A (the "prep" group) received mechanical bowel preparation with four administration of polyethylene glycol 12 to 16 hours before surgery, and Group B (the "non-prep" group) had no preoperative mechanical bowel preparation. All patients were allowed to have a regular diet until midnight the evening before surgery (patients in the prep group usually took their mechanical preparation after the last solid meal). All of the patients received perioperative broad-spectrum intravenous antibiotics (cephalosporine 2 g and metronidazole 500 mg b.i.d.), which were continued for at least 24 hours postoperatively. Surgeons were allowed to continue the prophylactic intravenous antibiotics for more then 1 day if necessary. 5 surgeons were enrolled in the study, all with high specialisation in colorectal resections (more than 20 procedure/year).

Patients undergoing rectal surgery were given one enema on the day before surgery to avoid extrusion of stool when using a transanally inserted stapling device.

All patients gave their informed consent before randomization in the study.

Data relative to patients' demographic and clinical characteristics, operative procedures and findings, and 30-day postoperative follow-up were prospectively entered in a Microsoft Excel database. The main outcome was the rate of postoperative infectious complications, such as wound infection, anastomotic leak, and intra-abdominal abscess. Wound infection was defined as a wound requiring partial or complete opening for drainage of purulent collection, or erythema requiring initiation of antibiotic treatment. Anastomotic leak was identified if demonstrated by imaging or documented in surgery, or if fecal drainage was evident through a perianastomotic drain. Abdominal abscess was defined as fluid collection demonstrated by computed tomography scan, in conjunction with elevated temperature or white blood cell count.

Statistical analysis was performed using the Fisher exact test or unpaired *t *test and probability values of less than 0.05 were considered significant (XLStat software).

## Results

Three hundred six patients were entered into the study between July 2005 and September 2009. Sixty-two patients were excluded after randomization due to the exclusion criteria (abdominoperineal resection, transanal resection for T1, TME with sphincter saving procedure after neo-adiuvant therapy for middle or low rectal cancer, R2-resection, randomisation in other studies, urgency or emergency procedures, patients who required a diverting stoma proximal to the anastomosis and those who were found to have an abdominal abscess at the time of surgery). One hundred twenty patients had their surgery with preoperative mechanical bowel preparation, while one hundred twenty-four did not have mechanical preparation. Demographic characteristics, type of surgery and type of anastomosis did not significantly differ between the two groups (Table 1).

**Table 1:** Demographics and clinical characteristics

	Prep (n:120)	Non-Prep (n:124)
*Mean Age (SD)*	71,3 (10.8)	69.8 (10.9)

*Gender*	120	124
Male	65	60
Female	55	64

*Surgical procedure*	120	124
Right colectomy	40	50
Transverse colectomy	9	4
Left colectomy	13	26
Sigmoidectomy	25	15
Anterior resection	33	29

*Localisation*	120	124
Colon	87	95
Rectum (upper)	23	29

*Staging*	120	124
Stage I	9	25
Stage II	52	34
Stage III	59	65

*Anastomosis*	120	124
Manual	70	88
Mechanical	50	36

The median length of postoperative antibiotic treatment was 2.7 (SD 0.8) days in the prep group and 2.7 (SD 0.7) days in the nonprep group (*P *= NS).

When assessing the main outcomes of this study, there was no significant difference in the rate of postoperative wound infections, clinical anastomotic leaks, or intra-abdominal abscesses between the prep and the non-prep group (Table 2). We found no difference in anastomotic leak with stratification for colonic and rectal surgery. The surgical infectious complications rate was 20.0% in the prep group and 11.3% in the non-prep group (p .05).

**Table 2:** Results: infectious complications

	Prep (n:120)	Non-Prep (n:124)	p-Value
*Wound infection*	**11 (9.2%)**	**6 (4.8%)**	**0.18**
*Anastomotic leakage*	**7 (5.8)**	**5 (4.0)**	**0.52**
*Colon*	**2**	**2**	**0.97**
*Rectum*	**5**	**3**	**0.44**
*Abdominal abscess*	**6 (5%)**	**3 (2.4)**	**0.36**
*Total*	**24 (20%)**	**14 (11.3)**	**0.05**

There was no significant difference in the average days to the first bowel movement and the length of hospital stay between the prep group and the non-prep group (4.9 days vs. 4.1 days, and 11.9 days vs. 11.0 days, respectively).

Mortality occurred in four patients in group A and two patients in group B (3.3% in the prep group, and 1.6% in the non-prep group). One patient in each group died due to sepsis from an anastomotic leak. Although none of these patients underwent an autopsy, none of the other four deaths was attributed to surgical infectious complications (2 cardiac, 1 respiratory, 1 neurologic disease).

## Discussion

Preparation for elective colon and rectal surgery with mechanical cleansing and antibiotic prophylaxis, in conjunction with improved surgical techniques and advances in perioperative care, served to reduce the rate of infectious complications in colorectal surgery. Although mechanical bowel preparation before elective colorectal surgery has become a surgical dogma, there is a paucity of scientific evidence demonstrating the efficacy of this practice in reducing the rate of infectious complications.

Whereas some animal studies have shown that mechanical preparation improved anastomotic bursting strength [16,17] and decreased septic complications, others failed to find a difference between groups of animals with or without bowel preparation [18]. Further evidence questioning the utility of mechanical bowel preparation in colorectal surgery comes from the literature regarding the management of urgent cases, such as patients with penetrating colonic trauma or acute colonic obstruction. In cases of penetrating trauma, prospective randomized studies have shown that primary colonic anastomosis is safe [19,20] even though the colon is not prepared, the mechanism of injury is not as controlled as in elective cases, and there is often a delay between the injury and the repair. These studies have led to a change in the standard of care of penetrating colonic trauma toward primary colonic repair é [14,15].

In cases of acute colonic obstruction, resection with primary anastomosis in one stage is not the common practice, as the colon is not prepared. Advanced techniques, such as on-table bowel lavage [21,22] or colonic metallic stents [23,24], have been used in an effort to allow mechanical bowel cleansing before primary anastomosis. Few authors, however, have challenged the dogma that colon resection with primary anastomosis is unsafe in patients with obstructing colon lesions. Few series suggested that anastomosis between the small bowel and the colon, as performed in right or subtotal colectomy, may be safe without mechanical preparation [25,26], since this type of anastomosis avoids the stool column proximal to the anastomosis. In a multicentric trial, [27] 97 patients with malignant left colonic obstruction were randomized to have either a segmental colon resection with on-table bowel lavage or a subtotal colectomy. The rates of intra-abdominal sepsis and anastomotic leaks did not significantly differ between the two groups. Other authors have suggested that colo-colonic anastomosis may also be safe in an unprepared bowel in the face of an obstructed colon é [25,28,29]. Recently, Naraynsingh et al. [30] reported a prospective series of 58 unselected patients with left colonic obstruction. All underwent segmental colon resection with primary colo-colonic anastomosis, without a proximal diverting stoma. There was one case of anastomotic leak and one mortality unrelated to infection.

Other published studies [31-34] have prospectively randomized patients undergoing elective colon and rectal surgery to having mechanical bowel preparation or no mechanical preparation. Although all of the prior studies are smaller in numbers then the current study, they also failed to show a benefit to mechanical bowel preparation in reducing the rate of infectious complications and anastomotic leaks.

Although the new agents used for mechanical bowel preparation such as polyethylene glycol and sodium phosphate are strong cathartic agents, the colon is frequently not completely clean and dry at the time of surgery. In our experience fluid or semifluid stool was often found in the patients of the prep group. When preparation is done for colonoscopy, liquid stool can be easily aspirated to provide adequate cleansing for a safe and effective colonoscopy. In contrast, when used as a preparation for surgery, it is more difficult to control liquid than solid stool, which may lead to the significantly higher rate of intraoperative spillage of contaminated bowel content. When mechanical bowel preparation is used, the use of a clear liquid diet before surgery, in conjunction with the cathartic agent, may potentially improve the quality of the preparation and reduce the rate of liquid colonic content.

Recently two studies [12,14] show no benefit of mechanical bowel preparation in elective colorectal resection and suggested that bowel preparation could be omitted before this type of surgery. And Bretagnol [13] says that avoid bowel preparation may be associated with reduced postoperative morbidity in elective rectal cancer surgery.

Finally a Cochrane review [15] that included a total of 13 RCTs (with 4777 participants: 2390 allocated to bowel preparation and 2387 to no preparation before elective colorectal surgery) concluded that there is no statistically significant evidence that patients benefit from bowel preparation.

Mechanical bowel preparation is not harmless. It almost invariably causes significant discomfort to the patient, including nausea, abdominal bloating, and diarrhea [4,6]. Mechanical bowel preparation is also associated with electrolyte imbalance and dehydration, [4,5] which may complicate the induction of anesthesia and perioperative care. Thus, in our view, mechanical bowel preparation should be treated as a medication and used only when indicated.

The results of this study strongly suggest that elective colon and rectal surgery may be safely performed without the use of routine mechanical bowel preparation. Bowel cleansing should therefore be used selectively for instance, in cases where intraoperative colonoscopy is likely to be required. The recent Cochrane review requires further research on patients submitted for elective colorectal surgery in whom bowel continuity is restored, with stratification for colonic and rectal surgery. In our experience, we not found differences in anastomotic leakage between groups in patients underwent at colon or rectal surgery, but further and larger studies are needed, also considering surgery of mid or low rectal cancer after neoadiuvant therapy.

## Competing interests

The authors declare that they have no competing interests.

## Authors' contributions

*SS*, surgeon and principal investigator, participated in surgical procedures, design and coordination of the study. *ER, ER, RS, GD, DP*, surgeons, partecipated in surgical procedures *VF*, chief of Surgical Oncologt Unit, partecipated in surgical procedures. All authors read and approved the final manuscript.
